The article "Efficacy of Human Umbilical Cord Blood-Mononuclear Cell Transplantation for MSA Treatment and Its Effects on Changes in T-Cell Subsets in Peripheral Blood and Inflammatory Factors" was published in 2021. Journal: Dis Markers.

# Efficacy of Human Umbilical Cord Blood-Mononuclear Cell Transplantation for MSA Treatment and Its Effects on Changes in T-Cell Subsets in Peripheral Blood and Inflammatory Factors

**DOI:** 10.1155/2021/5290766

**Published:** 2021-12-01

**Authors:** Haiyan Yu, Xiaoling Yuan, Min Zhao, Weifei Wang, Dianrong Gong

**Affiliations:** Department of Neurology, Liaocheng People's Hospital, Liaocheng, China

## Abstract

**Objective:**

This study is aimed at examining the efficacy of human umbilical cord blood-mononuclear cell (hUCB-MNCs) transplantation through lateral atlanto-occipital space puncture in multiple system atrophy (MSA) treatment and investigating changes in T-cell subsets in peripheral blood and inflammatory factors in patients before and after treatment.

**Methods:**

A total of 20 patients with MSA who underwent hUCB-MNC transplantation through lateral atlanto-occipital space puncture in the Liaocheng People's Hospital were enrolled. Patients were followed up at 0, 1, 3, and 6 months after treatment, and the Unified Multiple System Atrophy Rating Scale (UMSARS) scores, TNF-*α* in the peripheral blood, IL-6, percentage of CD4, and CD4/CD8 ratio were evaluated and compared for each follow-up point; any adverse effects were recorded.

**Results:**

UMSARS Part I scores were 20.55 ± 3.80, 19.20 ± 3.78, and 19.40 ± 4.11, 1, 3, and 6 months, respectively, after treatment and were significantly lower as compared to that before treatment (23.50 ± 4.72; *P* < 0.05). Similarly, UMSARS Part II scores 1, 3, and 6 months after treatment were 25.50 ± 5.01, 24.05 ± 5.01, and 24.25 ± 5.05, respectively, significantly lower as compared to that before treatment (30.15 ± 5.63; *P* < 0.05). The IL-6 values in the peripheral blood 1, 3, and 6 months after treatment were 5.25 ± 2.70 pg/m, 2.96 ± 1.75 pg/m, and 3.31 ± 1.62 pg/m, respectively, which were significantly lower (*P* < 0.05) than that before treatment (8.22 ± 4.69) pg/m. The TNF-*α* levels at 3 and 6 months after treatment were 13.08 ± 6.13 pg/m and 12.24 ± 4.76 pg/m, respectively, which were significantly lower than that before treatment (22.99 ± 13.30; *P* < 0.01). The CD4/CD8 ratios in the peripheral blood 1, 3, and 6 months after treatment were 1.09 ± 0.25, 1.30 ± 0.24, and 1.43 ± 0.22, respectively, which were significantly different than that before treatment (0.81 ± 0.24, *P* < 0.01). Similarly, the CD4 percentages 1, 3, and 6 months after treatment were 34.09 ± 1.79, 36.05 ± 1.50, and 36.47 ± 1.47, respectively, which were significantly different than that before treatment (0.81 ± 0.24; *P* < 0.01).

**Conclusion:**

hUCB-MNC transplantation through lateral atlanto-occipital space puncture could significantly improve the symptoms and signs in patients with MSA and delay the disease progression. Thus, hUCB-MNCs may modulate immune activity and reduce the inflammatory response.

## 1. Introduction

Multiple system atrophy (MSA) is a group of sporadic, maturity-onset, and neurodegenerative diseases with unknown etiology [1]. Clinically, MSA can be divided into the MSA-P type, where Parkinsonian syndrome is the prominent manifestation and the MSA-C type with cerebellar ataxia as the prominent manifestation. According to epidemiological statistics, the incidence rate of MSA in Europe and the United States is estimated at 0.6 per 100,000 people, with a prevalence rate of approximately 1.9~4.9 per 100,000 individuals [2]; among them, the MSA-P type predominates. In contrast, among the Chinese, the prevalence of MSA-C type dominates. However, complete epidemiological information from China at present is lacking. Overall, MSA progresses rapidly, and patients have a poor prognosis.

MSA pathology is characterised by the presence of immunoreactive glial cytoplasmic inclusions (GCIs) of the alpha-synuclein in microglia. Given that the cause and pathogenesis of MAS remain unknown, currently, there is no recognized treatment for the disease. Previous studies have emphasised the important role of neuroimmunity in the pathogenesis and progression of MSA, including changes in multiple immune cells, inflammatory factors, and chemotactic factors [3]. Clinical trials report improvements in symptoms and signs in MSA patients with intravenous immunoglobulin [4], suggesting underlying immune-mediated mechanisms in the pathogenesis of MSA. In this context, the relationship between immunology and degenerative diseases has become a current research hotspot.

After a decade of preliminary clinical trials, our group has reported good clinical outcomes [5–8] in the treatment of MSA, Parkinson's disease (PD), and delayed encephalopathy after acute carbon monoxide poisoning (DEACMP) by transplanting hUCB-MNCs through lateral atlanto-occipital space puncture (Gong's puncture method) into patients under the premise of safety and feasibility [9, 10]. However, the exact mechanism of action remains unclear.

8w?>In this study, hUCB-MNCs were transplanted through the lateral atlanto-occipital puncture to treat patients with MSA. The clinical data, immune function, and changes in inflammatory factors were evaluated, analysed, and summarised. The findings may provide a new direction for examining the pathogenesis and clinical management of MSA.

## 2. Materials and Methods

### 2.1. Materials

#### 2.1.1. Subjects

The study design was approved by the Hospital Ethics Committee (ID: 2019085), and informed consent was obtained from all subjects or their families.

Patients with MSA were enrolled from the Department of Neurology of the Liaocheng People's Hospital between April 2020 and April 2021 (all subjects met the revised clinical diagnostic criteria of 2008) and underwent hUCB-MNC transplantation through the lateral atlanto-occipital space puncture. Among them, 14 were males and six were females, with ages ranging from 44 to 71 years and a mean age of 55.4 ± 3.9 years. In addition, the disease duration of these patients ranged between 1.5 and 5 years, with a median duration of 2.7 ± 1.2 years. There were 17 patients with MSA-C and three patients with MSA-P types; 20 patients had autonomic dysfunction. The scoring method followed the *Unified Multiple System Atrophy Rating Scale* (UMSARS) established by the European Multiple System Atrophy Research Group in 2004 [11, 12]. The average UMSARS Part I and UMSARS Part II scores before treatment were 23.50 ± 4.72 points and 30.15 ± 5.63 points, respectively. Twenty patients showed varying degrees of cerebellar and brainstem atrophy as per their cranial magnetic resonance (MR) images. In three patients, the typical “hot cross bun sign” on the pons could be identified using MR T2WI images. Moreover, the shell nucleus fissure signs were observed in the T2WI images of another patient.

#### 2.1.2. Inclusion Criteria

According to the revised clinical diagnostic criteria for MSA, 2008, proposed by Gilman et al. [13], all included patients met the sporadic, progressive, and maturity-onset (over 30 years of age) characteristics of MSA. In addition, they also had the following characteristics.

*(1) Either One of the following*.

1. Levodopa malresponsive Parkinson's syndrome (bradykinesia accompanied by myotonia, tremors, or postural instability)
2. Cerebellar dysfunction (gait ataxia accompanied by cerebellar dysarthria, limb ataxia, or cerebellar oculomotor disorder)

*(2) At Least One of the following Autonomic Dysfunctions*.

1. Urinary incontinence (inability to control bladder urination combined with erectile dysfunction in men)
2. Postural hypotension (systolic blood pressure dropped ≥30 mmHg and/or diastolic blood pressure dropped ≥15 mmHg after 3 min of standing)

#### 2.1.3. Exclusion Criteria

Patients with (1) malignant tumours; (2) active tuberculosis or serious uncontrolled infectious diseases; (3) serious organic diseases of the heart, liver, kidney, or other organs; (4) mental illness; (5) serious blood disorders or coagulation disorders; or/and (6) allergies were excluded from this study.

### 2.2. Methods

1. The pretreatment procedures included routine blood examination, erythrocyte sedimentation rate evaluation, full biochemical test, whole-body tumour marker-based screen, viral screen, coagulation tests, chest CT, cranial MR, serum interleukin assay, and T cell subset and count evaluation
2. Preparation of hUCB-MNCs: the cord blood was provided by the Obstetrics Department of the Liaocheng People's Hospital (negative for hepatitis B, hepatitis C, AIDS, syphilis, and other relevant infectious indicators) and approved by the Hospital Ethics Committee for ethical compliance. The hUCB-MNCs were isolated and extracted by professionals in the Central Laboratory of our Hospital using a cord blood processing kit (developed by Wilson Canada, manufactured by Ningxia Zhonglianda Biological Co., Ltd., specification: SCR-200I). Briefly, 5 mL of hUCB-MNC suspension [(2 ~ 3) × 108/mL] was obtained. The cells were tested and those with viability ≥ 98% were immediately delivered to the ward in a cryogenic transport box at 0°C~4°C. These were transplanted into patients within an hour after rewarming
3. Injection of hUCB-MNCs: the hUCB-MNCs were injected through the lateral atlanto-occipital space puncture method [5]. Specifically, the patient laid flat with his head in the middle of the operating table and neck straight. The injection site was 1 cm below and behind the highest point of the mastoid process. After routine disinfection and local anaesthesia, the puncture needle was placed parallel to the hypothetical line of the external auditory canal and perpendicular to the longitudinal axis of the cervical vertebra. The needle was then inserted along the inferior border of the occipital bone. Under normal conditions, patients would experience falling sensations twice during the puncture. The puncture was considered successful if there was a breakthrough sensation, cerebrospinal fluid flow on the removal of the stylet, and immediate access to the cisterna magna. Next, 3 mL of cerebrospinal fluid was retained for examination. 5 mL of rewarmed hUCB-MNCs was slowly injected into the cisterna magna. Subsequently, the puncture needle was removed; the puncture site was pressed and covered with a sterilized dressing. The procedure was strictly aseptic, and the patient was placed in a decubitus position for 6-8 hours. Each patient underwent the treatment thrice at one-month intervals
4. Serum interleukin assay of the peripheral blood and T-cell subset and count examinations were performed by the Central Laboratory of Liaocheng People's Hospital, followed by the issuance of a test report

#### 2.2.1. Evaluation Method

1. Blood routine examination, hepatorenal function tests, tumour marker-based screening, and viral screen were performed to detect possible adverse reactions
2. Patients were followed up 1, 3, and 6 months after their first hUCB-MNC transplantation treatment. Their UMSARS scores, TNF-*α* levels, IL-6 levels, CD4%, and CD4/CD8 ratios were compared at each follow-up point

### 2.3. Statistical Analysis

Clinical data were analysed using the SPSS 26.0 statistical software (IBM SPSS Statistics for Windows) and expressed as mean ± standard deviation. Analysis of variance (ANOVA) for repeated measurements was used to compare the data at multiple time points before and after treatment, where two-by-two comparisons at each time point were performed using the Bonferroni test. Differences with *P* < 0.05 were considered statistically significant.

## 3. Results

### 3.1. Safety

Three patients reported a mild headache on the first-day posttreatment, but their symptoms disappeared completely within three days of sufficient rest and hydration with water. One patient developed a slight fever on the second-day posttreatment, with a maximum body temperature of 37.5°C; however, there were no significant abnormalities upon blood examinations, and the body temperature was normal within 12 hours after symptomatic treatment without recurrence. The remaining patients did not report any discomfort. Continuous cardiac monitoring was performed for 24 hours after treatment, and vital signs were stable in all patients. Laboratory tests, including blood, urine, and stool routine examinations, hepatorenal function tests, tumour marker-based screens, and viral screens were performed at 1-, 3-, and 6-month follow-up after treatment. These showed no significant differences as compared to the levels before treatment. No tumours were found in chest CT. In patients with preexisting lung nodules, there was no increase in the nodule size. Additionally, no other transplant-related complications emerged within six months of follow-up posttreatment.

### 3.2. Effects of hUCB-MNC Transplantation through Lateral Atlanto-Occipital Space Puncture on UMSARS Part I and Part II Scores in MSA Patients

The results of ANOVA for repeated measurements showed significant differences in UMSARS Part I and UMSARS Part II scores at different follow-up time points (*P* < 0.05). Compared to the scores before treatment, the UMSARS Part I scores and the UMSARS Part II scores decreased significantly 1, 3, and 6 months after treatment as compared to that before treatment (*P* < 0.05). In two-by-two comparisons at different time points after treatment, no statistically significant differences between the UMSARS Part I and Part II scores were observed (*P* > 0.05). The above results are summarized in Table 1.

### 3.3. Effects of hUCB-MNC Transplantation through Lateral Atlanto-Occipital Space Puncture on Immune Function and Inflammatory Factors

1. The results of ANOVA for repeated measurements showed significant differences in IL-6 and TNF-*α* values at different times (*P* < 0.05). IL-6 values were significantly lower at 1, 3, and 6 months after treatment as compared to that before treatment (*P* < 0.05); TNF-*α* values were significantly lower at 3 and 6 months after treatment as compared to that before the transplant (*P* < 0.05). However, there were no statistically significant differences in two-by-two comparisons at different time points after treatment (*P* > 0.05). The decrease in the proinflammatory factors suggested a reduced inflammatory response after treatment. The above results are summarized in Table 2

(2) The results of ANOVA for repeated measurements showed significant differences in CD4 percentages and CD4/CD8 ratios at different follow-up time points (*P* < 0.05). The CD4 percentages and CD4/CD8 ratios were significantly higher at all time points after treatment as compared to corresponding values before treatment (*P* < 0.05). The differences in CD4 percentages and CD4/CD8 ratios were significant (*P* < 0.05) at 3 and 6 months after treatment as compared to corresponding values 1 month after treatment, which suggested alterations in cellular immune functions. The above results are summarized in Table 3

## 4. Discussion

MSA is an insidious disease associated with a rapid progression and poor prognosis. To date, available therapeutic options for MSA remain inadequate. Several preclinical studies illustrate the roles of cell transplantation in neuroprotection, neural restoration, improvement of the brain environment, and immune modulation. In this context, relevant clinical trials have been conducted in recent years. In late 2017, the US-FDA approved an expanded clinical scope for cord blood cell therapy in the treatment of several diseases, including cerebral palsy, autism, and cerebral ischemia, thereby, providing effective cord blood therapy options for more patients with neurological disorders. The hUCB-MNCs used in this study have the following advantages: (1) they are derived from umbilical cord blood discarded at delivery, thereby, are noninvasive and ethically uncontroversial; (2) they are available from adequate sources, and the isolation and collection are easy; (3) they are safe to use, owing to the primitive nature of their immune system and low antigenicity.

The hUCB-MNCs extracted from cord blood consist of a mixed cell population, including stem cells, endothelial progenitor cells, regulatory T cells, natural killer cells, T lymphocytes, and dendritic cells. These cells actively play a protective role in the progression of neurodegenerative diseases [14]. The hUCB-MNCs can self-renew, proliferate, differentiate, as well as induce differentiation. Notably, it also exerts paracrine effects; its secreted exosomes, growth factors, and cellular immune factors exhibit immunomodulatory effects without major histocompatibility complex (MHC) restriction [15]. Therefore, its use in neurodegenerative diseases, degenerative diseases, and immunological diseases has received increasing attention.

In clinical settings, hUCB-MNC transplantation is performed by various methods, including intravenous injection, lateral ventricular puncture, lumbar puncture, and stereotactic techniques. The lateral atlanto-occipital space puncture was invented by Prof. Gong Dianrong in 1996; it is complementary to the lumbar puncture technique and is used in clinical treatment [9]. Since 2011, our group, by combining lateral atlanto-occipital gap puncture with hUCB-MNC transplantation, has successfully injected cells directly into the cerebellomedullary cistern. To date, more than 700 treatments for over 400 cases, spanning across more than 20 refractory neurological diseases, have been performed, safely and effectively [10]. Lateral atlanto-occipital space puncture is a very effective method for cell transplantation, owing to its high success rate, broad applicability, minimal trauma, short operation time, and proximity of the injected cells to the lesion.

In this study, hUCB-MNCs were transplanted through lateral atlanto-occipital space puncture into 20 patients with MSA. According to the data, the UMSARS scores after treatment declined significantly during the six-month follow-up period, and there were significant improvements in neurological functions and patients' quality of life, which further proved the safety and efficacy of this treatment procedure.

The specific pathological changes in MSA are associated with the presence of GCIs within the cytoplasm of oligodendrocytes, with alpha-synuclein as the main component. According to the present findings, both microglia and immune-related T lymphocytes could be involved in the abnormal clustering of alpha-synuclein, and the subsequent formation of GCI may trigger a series of inflammatory immune responses, eventually leading to neuronal cell degeneration and necrosis [2, 16–18]. Animal studies show apoptosis and immune activation in the pathogenesis of neurodegenerative diseases. Bas et al. report an imbalance in T-cell subsets in the peripheral blood of patients with Parkinson's disease, which was mainly manifested due to reduced CD4+ percentages and CD4/CD8 ratios [19, 20]. As an important indicator of the immune response, changes in lymphocyte subsets in the peripheral blood of MSA patients deserve further clinical attention.

T lymphocytes can cross the blood-brain barrier and influence the progression of neurodegenerative diseases [21]. In addition, T lymphocytes are involved in body-specific immune responses. CD4 exerts an anti-infective immune effect, and CD8 is involved in cytotoxic responses. The levels of several T cell-related cytokines were altered in the body fluids of patients with MSA, which suggested that cell-mediated immunity was involved in the progression of MSA. Changes in T cell subsets are also associated with the progression of MSA. Researchers have identified the interaction of microglia with CD4+ T cells and alpha-synuclein in the *in vitro* models. Regulatory T cells suppress alpha-synuclein-induced oxidative stress, while effector T cells exacerbate microglia inflammation and induce neurotoxic responses [22]. hUCB-MNC, in addition to their regenerative function, can function as immunomodulators through the secretion of the mesenchymal stem cell-derived exosomes. After injecting these secretions into the substantia nigra and striatum of the animal model for the disease, an increase in the dopaminergic neurons in the brain and an improvement in the motor behaviour of the experimental animals were observed [23]. *In vitro* studies show that hUCB-MNC can inhibit the proliferation of T cells, induce apoptosis of activated T cells, suppress the proliferation of B cells, inhibit the cytotoxic effects of CTLs, and alter the TH1/TH2 balance [15]. In addition, foreign studies show that immunotherapy may be effective for patients with MSA [24].

As important mediators of the immune responses, cytokines influence every process of the inflammatory response cascade. High expression of several proinflammatory cytokines and chemokines, including TNF-alpha, MCP, IL-6, and IL-1, have been found in brain tissues from autopsies of patients with neurodegenerative diseases such as PD and MSA [25, 26], suggesting that these cytokines are involved in the progression of MSA. Findings from the *in vitro* models demonstrate that alpha-synuclein induces apoptosis of neurons, proliferation of microglia, and secretion of the tumour necrosis factor, TNF-alpha [27]. Therefore, it can be reasonably hypothesized that alpha-synuclein activates the immune system, leading to the production of cytokines, chemokines, and the complement system. Li et al. [28] performed immunohistochemical staining of brain tissues from postmortem pathologically confirmed MSA patients and found that alpha-synuclein deposition was substantially associated with significant upregulation of inflammatory cells and neurodegenerative processes. Experimental studies in animals show that implantation of modified MSCs reduces the release of TNA-alpha and interleukins to suppress the immune-inflammatory response and enhance the proliferation of astrocytes. Thereby, astrocytes may influence the survival time of neurons through relevant immune-inflammatory pathways [29]. After four weeks following intravenous injection of MSCs in a mouse model of MSA, Stemberger et al. [30] found significant reductions in levels of IL-1, IL-2, IL-6, IL-17, and TNF-alpha, inhibition of inflammatory immune responses, reduction in astrocyte and microglia activation in the brains of MSA animals, and recovery in the total number of TH+ neurons in the substantia nigra pars compacta (SNC) [30, 31].

Our results showed abnormal values of inflammatory cells and T-lymphocyte subsets in peripheral blood of patients with MSA. However, as their conditions improved, CD4 values and CD4/CD8 ratios increased, along with a concomitant decrease in inflammatory cytokines, IL-6 and TNF-alpha levels, which suggested that hUCB-MNCs could alter the imbalance of T-cell subsets, modulate the cellular immune responses, and suppress the inflammatory responses in patients with MSA.

In summary, a relationship between cellular immune disorders and inflammatory responses and MSA was observed. hUCB-MNCs may function by inhibiting T lymphocyte proliferation and downregulating inflammatory factors associated with T cell subsets, inflammatory cytokine and microglial activation, glial cell proliferation, and adaptive immune regulation. hUCB-MNCs contain haematopoietic stem cells, MCs, endothelial progenitor cells, and T lymphocytes. Thus, hUCB-MNCs can differentiate and replace damaged neuronal cells. In addition, with the help of its immune cells and paracrine cytokines, hUCB-MNCs can modify the pathogenic microenvironment, suppress the inflammatory responses, and modulate the immune responses in MSA patients [14].

Our study demonstrated the safety and efficacy of hUCB-MNC transplantation through lateral atlanto-occipital space puncture for the treatment of MSA. In addition, hUCB-MNC may function by modulating the immune responses and reducing the inflammatory responses. The results of this study may provide a reference for investigating the role of immune-inflammatory responses in the progression of MSA and provide theoretical support and therapeutic strategy development direction for hUCB-MNC transplantation in the treatment of neurodegenerative diseases, such as MSA. However, our study is a single-center small sample study. Thus, we would continue to identify novel markers to achieve breakthroughs in the treatment of MSA.

## Figures and Tables

**Table 1:** UMSARS Part I and II scores before and after treatment.

Indicator	*N*	Value before treatment	Values after treatment			*F* value	*P* value
			1 month	3 months	6 months		
UMSARSI	20	23.50 ± 4.72	20.55 ± 3.80^a^	19.20 ± 3.78^a^	19.40 ± 4.11^a^	4.634	0.005
UMSARSII	20	30.15 ± 5.63	25.50 ± 5.01^a^	24.05 ± 5.01^a^	24.25 ± 5.05^a^	5.596	0.001

^a^Significant difference compared to values before treatment (*P* < 0.05).

**Table 2:** Laboratory values of inflammatory factors before and after treatment.

Indicator	*N*	Value before treatment	Values after treatment			*F* value	*P* value
			1 month	3 months	6 months		
IL-6 (pg/mL)	20	8.22 ± 4.69	5.25 ± 2.70^a^	2.96 ± 1.75^a^	3.31 ± 1.62^a^	13.271	0.0001
TNF-*α* (pg/mL)	20	22.99 ± 13.30	17.04 ± 8.75	13.08 ± 6.13^a^	12.24 ± 4.76^a^	6.145	0.0008

^a^Significant difference compared to values before treatment (*P* < 0.05).

**Table 3:** CD4 percentages and CD4/CD8 ratios before and after treatment.

Indicator	*N*	Value before treatment	Values after treatment			*F* value	*P* value
			1 month	3 months	6 months		
CD4/CD8	20	0.81 ± 0.24	1.09 ± 0.25^a^	1.30 ± 0.24^ab^	1.43 ± 0.22^ab^	25.78	0.0001
CD4%	20	31.31 ± 1.89	34.09 ± 1.79^a^	36.05 ± 1.50^ab^	36.47 ± 1.47^ab^	39.66	0.0001

^a^Significant difference compared to values before treatment (*P* < 0.05); ^b^significant difference compared to values 1 month after treatment (*P* < 0.05).

## Data Availability

The data used to support the findings of this study are available from the corresponding author upon request.

## References

[1] Jianping J., Shengdi C. (2018). *Neurology*.

[2] Wenning G. K., Colosimo C., Geser F., Poewe W. (2004). Multiple system atrophy. *Lancet Neurology*.

[3] Jellinger K. A., Wenning G. K. (2016). Multiple system atrophy: pathogenic mechanisms and biomarkers. *Journal of Neural Transmission*.

[4] Novak P., Williams A., Ravin P., Zurkiya O., Abduljalil A., Novak V. (2012). Treatment of multiple system atrophy using intravenous immunoglobulin. *BMC Neurology*.

[5] Weifei W., Haiyan Y., Xiaoling Y. (2020). And other clinical studies of umbilical blood mononuclear cells for the treatment of Parkinson's disease. *Journal of Chinese Cell and Stem Cell*.

[6] Dianrong G., Haiyan Y., Min Z., Xiaoling Y., Qian L. (2016). Clinical observation of umbilical blood mononuclear cells in lateral occipital space for multisystemic atrophy. *Journal of Chinese Cell and Stem Cell*.

[7] Dianrong G., Haiyan Y., Qian L. (2013). Subarachnoid transplantation of umbilical blood mononuclear cells for late encephalopathy after carbon monoxide poisoning. *Journal of Chinese Cell and Stem Cell*.

[8] Gong D., Yu H., Wang W., Yang H., Han F. (2013). Human umbilical cord blood mononuclear cell transplantation for delayed encephalopathy after carbon monoxide intoxication. *Journal of Neurosurgery*.

[9] Gong D., Yu H., Yuan X. (2018). A new method of subarachnoid puncture for clinical diagnosis and treatment: lateral atlanto-occipital space puncture. *Journal of Neurosurgery*.

[10] Yu H., Gong D., Yuan X. (2018). Analysis of the efficacy of human umbilical cord blood mononuclear cells in refractory neurological diseases by lateral puncture of the global occipital space. *Chinese Journal of Cell and Stem Cell (Electronics)*.

[11] Wenning G. K., Tison F., Seppi K. (2004). Development and validation of the Unified Multiple System Atrophy Rating Scale (UMSARS). *Movement Disorders*.

[12] Weihong G., Guoxiang W. (2007). Multisystem atrophy scale assessment. *Chinese Journal of Neurology*.

[13] Gilman S., Wenning G. K., Low P. A. (2008). Second consensus statement on the diagnosis of multiple system atrophy. *Neurology*.

[14] Chen N., Hudson J. E., Walczak P. (2005). Human umbilical cord blood progenitors: the potential of these hematopoietic cells to become neural. *Stem Cells*.

[15] Phinney D. G., Pittenger M. F. (2017). Concise review: MSC-derived exosomes for cell-free therapy. *Stem Cells*.

[16] Yoshida M. (2007). Multiple system atrophy: *α*-synuclein and neuronal degeneration. *Neuropathology*.

[17] Song Y. J., Lundvig D. M., Huang Y. (2007). p25*α* Relocalizes in Oligodendroglia from Myelin to Cytoplasmic Inclusions in Multiple System Atrophy. *The American Journal of Pathology*.

[18] Yazawa I., Giasson B. I., Sasaki R. (2005). Mouse Model of Multiple System Atrophy *α*-Synuclein Expression in Oligodendrocytes Causes Glial and Neuronal Degeneration. *Neuron*.

[19] Bas J., Calopa M., Mestre M. (2001). Lymphocyte populations in Parkinson's disease and in rat models of parkinsonism. *Journal of Neuroimmunology*.

[20] Fiszer U., Piotrowska K., Korlak J., Członkowska A. (1991). The immunological status in Parkinson's disease. *Medical Laboratory Sciences*.

[21] Wilson E. H., Weninger W., Hunter C. A. (2010). Trafficking of immune cells in the central nervous system. *Journal of Clinical Investigation.*.

[22] Reynolds A. D., Stone D. K., Mosley R. L., Gendelman H. E. (2009). Nitrated *α*-Synuclein-Induced alterations in microglial immunity are regulated by CD4+T cell subsets. *Journal of Immunology*.

[23] Teixeira F. G., Carvalho M. M., Panchalingam K. M. (2017). Impact of the secretome of human mesenchymal stem cells on brain structure and animal behavior in a rat model of Parkinson’s disease. *Stem Cells Translational Medicine*.

[24] Shiraishi W., Iwanaga Y., Yamamoto A. (2015). A case of an anti-Ma2 antibody-positive patient presenting with variable CNS symptoms mimicking multiple system atrophy with a partial response to immunotherapy. *Rinsho Shinkeigaku Clinical Neurology*.

[25] Mogi M., Harada M., Riederer P., Narabayashi H., Fujita K., Nagatsu T. (1994). Tumor necrosis factor-*α* (TNF-*α*) increases both in the brain and in the cerebrospinal fluid from parkinsonian patients. *Neuroscience Letters*.

[26] Mogi M., Harada M., Kondo T. (1994). Interleukin-1*β*, interleukin-6, epidermal growth factor and transforming growth factor-*α* are elevated in the brain from parkinsonian patients. *Neuroscience Letters*.

[27] Zhang L. J., Ma P. J., Guan Q. K. (2018). Effect of chemokine CC ligand 2(CCL2) on a synuclein induced microglia proliferation and neuronal apoptosis. *Molecular Medicine Reports*.

[28] Li F. Z., Ayaki T., Maki T., Sawamoto N., Takahashi R. (2018). NLRP3 inflammasome-related proteins are upregulated in the putamen of patients with multiple system Atrophy. *Journal of Neuropathology and Experimental Neurology*.

[29] Xian P., Hei Y., Wang R. (2019). Mesenchymal stem cell-derived exosomes as a nanotherapeutic agent for amelioration of inflammation-induced astrocyte alterations in mice. *Theranostics*.

[30] Stemberger S., Jamnig A., Stefanova N., Lepperdinger G., Reindl M., Wenning G. K. (2011). Mesenchymal stem cells in a transgenic mouse model of multiple system atrophy: immunomodulation and neuroprotection. *PLoS One*.

[31] Stefanova N., Reindl M., Neumann M., Kahle P. J., Poewe W., Wenning G. K. (2007). Microglial activation mediates neurodegeneration related to oligodendroglial *α*-synucleinopathy: implications for multiple system atrophy. *Movement Disorders*.

